The article "Vocational Therapy of Physical Training for Children's Learning Motivation and Psychological Cognition" was retracted in 2024. Reasons: signs of a paper mill; suspected computer-generated content; unreliable results or conclusions; lack of ethics approval or compliance.

# Vocational Therapy of Physical Training for Children's Learning Motivation and Psychological Cognition

**DOI:** 10.1155/2022/8625830

**Published:** 2022-06-30

**Authors:** Geng Du, Tao Tao

**Affiliations:** ^1^Sports Training Department, Wuhan Sports University, Wuhan, Hubei 430079, China; ^2^School of Physical Education and Sports, Beijing Normal University, Beijing 100875, China

## Abstract

Childhood is an essential length for the formation and improvement of people's quite a number of psychological abilities; however, due to the damaging consequences of heredity, disease, surroundings, and education, it will carry poor outcomes to the ordinary improvement of kid's psychology. Good body satisfactory and wholesome psychology are vital which ensure to adapt to social competition. Carrying out suitable body exercise can decorate students' horrible psychological conditions, alter kid's negative emotions, promote students' intellectual enchantment, and enhance students' willpower. This paper researches the relationship between kid's gaining knowledge of motivation and psychological cognition and sports activity education occupational therapy, tries to discover out the influence of kid's studying motivation and psychological cognition on kid's sports activity coaching occupational therapy, analyses kid's sports coaching motivation from inside causes, and focuses on how to make college students extra inclined from controlling motivation to self-sustaining motivation, so that college students are inclined to take part in finding out about sports activities and structuring a robust activity in body education.

## 1. Introduction

Childhood is in a length of speedy body and intellectual development. It is a top time to domesticate true activity in body schooling and stimulate the motivation of body schooling learning, so as to lay a proper basis for students' lifelong body schooling and promote the healthful improvement of students' body and intellectual fitness [1]. Sports education occupational remedy can enhance the self-feeling capability of whole-body movement. Through sports activity ability education and physique cognizance exploration, it can amplify a range of emotional law and psychological characteristic improvement. Through different training, it can substantially promote kid's conversation capacity with others and then obtain the institution of kid's self-consciousness. According to the qualities of kid's body and mental development, body teaching occupational treatment is a purposeful rehabilitation-instructing endeavor for kids by way of precise plans with superb body schooling techniques as auxiliary techniques [2]. At present, there are many techniques of body coaching for orphans, and exact effects have been performed in some aspects. However, in rehabilitation training, some mothers and fathers and instructors frequently bypass the enchantment of kid's social verbal exchange ability; however, the focal point is on the education of language or feeling. In addition, the structure is single and the content material is boring, so that kid's enthusiasm is no longer high; they are now not fascinated in the content and cannot reap the predicted rehabilitation effect, which subsequently leads to the ineffective enchantment and enchantment of kid's social conversation ability. Due to kid's very own obstacles, they have been addicted to their very own world for a lengthy time, ensuing in a serious lack of social conversation ability, unable to adapt to the society, combine into the society, and even unable to live on and increase in the society [3]. Therefore, we ought to research about greater training modes and schooling strategies to decorate their social verbal change ability, save childhood from their very personal world, and make them adapt to the society and mix into the society as shortly as possible, which is of top-notch magnitude to the enchantment of the entire society.

The article "Vocational Therapy of Physical Training for Children's Learning Motivation and Psychological Cognition" was retracted in 2024. Reasons: signs of a paper mill; suspected computer-generated content; unreliable results or conclusions; lack of ethics approval or compliance.

Reveal the improvement vogue of kid's sports activity motivation and the degree of sports activity participation interest, so as to furnish theoretical foundation and reference hints for future sports activity teaching. In addition, analyse and talk about the relationship between sports activity participation hobby and sports activity motivation, give an explanation for the elements affecting kid's sports activities getting to know activity with one-of-a-kind dimensions, discover the interplay between kid's sports activity motivation and interest, and deeply recognize the software of self-determination idea in college body education. Therefore, most of its lookup is catered having an effect on exclusive sorts of motivation on behaviour and its impact [4]. In current years, a massive quantity of research is seemed to have specific fields, such as college education, household education, body training, psychotherapy, agency and management, and pal relationship. This research observes the effectiveness of self-sustaining motivation in merchandising people's fine behaviour [5]. From the lookup on the relationship between kid's sports activities mastering pastime and controlling motivation and independent motivation, this paper tries to locate out the effect on distinct two types of motivation on kid's sports activity gaining knowledge of interest, analyse kid's sports activity motivation from inner factors, know how to make university college students more inclined to self-sufficient motivation from controlling motivation, make university college students inclined to take section to locate out sports activity things to do matters and form a sturdy exercise in sports activity things to do learning, and adhere to body exercise for a prolonged time.

The article "Vocational Therapy of Physical Training for Children's Learning Motivation and Psychological Cognition" was retracted in 2024. Reasons: signs of a paper mill; suspected computer-generated content; unreliable results or conclusions; lack of ethics approval or compliance.

Different sorts of body exercise can promote a range of cognitive features of quite a number of groups, and the associated physiological mechanisms have been studied at exceptional levels. At the micro level, physical exercise is conducive to the dietary supply and energy metabolism of talent cells and can promote the survival of neurons and synapse formation. At the macro level, body workout can now not solely enhance the quantity of talent buildings such as the hippocampus and cerebellum, but additionally has an effect on the activation stage of intelligence areas and the useful connection of genius regions. Based on this, this paper intends to begin with the aggregation of sports activity education and occupational remedy training principle and practice, pays interest to the possible educating exercise in particular fixing kid's intellectual fitness problems, talks about how to enhance kid's intellectual fitness via sports activity educating reform, additionally furnishes a theoretical groundwork for enhancing the greatness of sports activity instructing and kid's intellectual fitness level, and puts forward sports activity education occupational remedy for kid's mastering motivation and psychological cognition. The organizational structure of this paper is as follows: Section 1 is the introduction, which introduces the relevant background, research significance, and the main work of this paper. Related work is discussed in Section 2.  Section 3 analyses the relevant theories and technologies. The experiment and analysis are carried out in Section 4.  Section 5 summarizes the full text.

## 2. Related Work

In latest years, the lookup on body exercise and kid's intellectual fitness has steadily increased, and the lookup in this discipline has made terrific progress. All educators beef up the lookup on the effect of body workout on students' intellectual fitness and its mechanism, which can supply scientific and nice education when college students take part in body exercise, and assist college students provide full play to the position of body exercise in regulating mental health, so as to assist enhance students' intellectual health. The applicable lookup is on the whole as follows:

Sports professional remedy is an organized, conscious and purposeful teaching and guiding career formed through a variety of organizational forms according to the physical and psychological improvement characteristics of children, with dreamlike physical exercise as the auxiliary ability[6]. At present, sports activity things to do training occupational treatment is substantially used in a range of instructing processes and is moreover used as an auxiliary capability for the treatment of wonderful children. Starting from the features of sports, some students have carried out relevant search for on the relationship between sports activity things to do and kid's mental health. In the face of an increasing number of extreme kid's intellectual fitness problems, some humans of perception in the present-day tutorial circles have carried out applicable lookup [7]. It can even be stated that the lookup on kid's intellectual fitness has been fruitful. However, most of this research are from the viewpoint of psychology, pedagogy, and sociology and have little contact with modern-day body schooling [8]. With the complete improvement of cultural best schooling in schools, the relationship between people's all-round improvement and college body schooling has additionally obtained due attention. Physical training has been included into the complete cultivation of people's great [9]. Around such a topic, many college students have moreover carried out affluent look up from a couple of tiers and angles, which has laid the foundation for the look up of this topic.

The article "Vocational Therapy of Physical Training for Children's Learning Motivation and Psychological Cognition" was retracted in 2024. Reasons: signs of a paper mill; suspected computer-generated content; unreliable results or conclusions; lack of ethics approval or compliance.

Some achievements have been made in finding children's intellectual health and physical education. However, unfortunately, the interaction between physical training and children's intellectual health education has been neglected because physical education is usually related to the cultivation of students' healthy physique for a long time [10]. Of course, as noted above, some college students are concerned about the greater and greater serious mental health problems of university college students in trendy schools and are combined with body training to a certain extent in the research; then again, it is highly insufficient. Moreover, by using the applicable search conducted by most students, this paper theoretically expounds the relationship between physical education and children's intellectual health training, which is distinctly easy even if there is the mixture of idea and practice; there is a relative lack of concrete and viable optimistic opinions [3, 11]. With the emergence of increasingly more extreme kid's intellectual fitness problems, how to domesticate awesome abilities with precise body and intellectual fitness in university schooling and overcome kid's psychological boundaries has turn out to be an extreme concern that university schooling cannot pass by [12]. Due to the late start of intellectual fitness schooling in China, intellectual fitness training is a complicated dynamic process; greater and extra youngsters go through from intellectual diseases, which influences the cultivation of excellent talents. Although there is nevertheless many research on the impact of body schooling on kid's intellectual health, most of this research are primarily based on pure theoretical research, much less grasp from the peak of body training idea and practice, vulnerable operability, and negative implementation impact [13].

The article "Vocational Therapy of Physical Training for Children's Learning Motivation and Psychological Cognition" was retracted in 2024. Reasons: signs of a paper mill; suspected computer-generated content; unreliable results or conclusions; lack of ethics approval or compliance.

## 3. Related Theories and Technologies

### 3.1. Micro Mechanism of Physical Training Promoting Cognitive Function

At the micro level, the acquisition of diet and the utilization of electricity are the integral conditions for neurons to raise out lifestyle's activities. On the foundation of ample diet grant and steady metabolism of energy, cells will correct the entire number of biochemical reactions and synthesize neurotransmitters, proteins, and different elements quintessential for neuron survival and synaptic establishment. Physical workout can have an effect on the above phone exercise technique [14]. For example, the lookup of brain-derived neurotrophic issue suggests that body exercise can have an effect on the biochemical response in cells, while the lookup associated with vascular merchandising and talent illnesses suggests that body exercise can have an effect on the vitamin grant and strength metabolism of cells. Brain-derived dietary elements play a promotion position in the manner of body exercise merchandising cognitive ability.

Physical workout can promote vascular fitness and make bigger cerebral blood flow, and enhance intelligence plasticity while bringing adequate vitamin and strength to the genius [15]. Morphological and anatomical studies showed that compared with the non exercise group, the cerebral cortical vessels in the exercise group were larger. Physical exercise can promote talent angiogenesis, enhance the dietary grant and strength metabolism of genius cells, and eventually enhance genius plasticity. However, it is really worth noting that angiogenesis cannot utterly provide an explanation for the complete mechanism of body exercise merchandising cognitive characteristics [16]. The lookup indicates that though patience coaching can at once enhance the fitness stage of blood vessels, low-intensity workout routines such as stretching coaching and coordination coaching can additionally promote cognitive function. The role model of physical training in promoting cognitive function is shown in Figure 1.

### 3.2. Effect of Physical Training and Occupational Therapy on Children's Psychological Cognition

In the fierce getting to know competition, students' mastering duties are usually heavy, so most college students will have some terrible emotions, such as anxiety, boredom, and melancholy in the system of learning. If students' horrific thoughts are no longer improved, over time, students' intellectual fitness will have problems, ranging from affecting their learning about lifestyles to inflicting some body illnesses [17, 18]. Therefore, we need to pay interest to the mitigation and law of students' terrible emotions. Through body exercise, it can assist college students launch their terrible thoughts and free themselves from terrible emotions, so that they can face the fierce studying opposition and heavy getting to know duties with an extra advantageous and fuller mindset [19].

The article "Vocational Therapy of Physical Training for Children's Learning Motivation and Psychological Cognition" was retracted in 2024. Reasons: signs of a paper mill; suspected computer-generated content; unreliable results or conclusions; lack of ethics approval or compliance.

In ordinary body education, we accept as true with that body workout can enhance students' body excellence and workout students' physique [20]. Students' strengthening body exercise can now not solely advance their intelligence, but additionally enhance their body quality. When college students take body exercise, they can promote the improvement and use their intelligence and assist and beautify their frightened device feature [21]. If the students' brain can be entirely developed, college students will no longer experience a task so challenging when finishing other mastering tasks, which helps to assist college students get rid of heavy mastering tasks, so as to enhance students' learning efficiency. In the true learning about life, college students have to have desirable social adaptability and harmonious interpersonal relationship, which is very necessary for the ordinary conversation between college students and others [22]. Many lookups have confirmed that remarkable body exercise can aid and beautify students' interpersonal relationships and decorate students' social adaptability. For students, body exercise is now no longer fully a body activity, then again moreover a social activity. Because in the method of body exercise, college students can speak with every different and be aware of extra new friends, so as to assist and beautify their capacity to adapt to society and others [23]. In the system of speaking with new friends, it can additionally assist college students launch their body and intellectual strain and promote their body and intellectual health. Steps and processes of physical training and occupational therapy are shown in Figure 2.

Only with a sturdy will can they have the braveness to overcome all the difficulties they encounter. During body exercise, college students can mood their will, due to the fact that in the technique of exercise, centre students will face some difficulties, while overcoming these difficulties, their will has additionally been increased [24]. For example, college students need to move all boundaries in front of them to the entire exercise when they are sprinting and hurdling. In the manner of hurdles, college students can tame their fighting spirit and strong will, so as to unite to overcome the difficulties they face every day [25]. Now college students are dealing with terrific gaining knowledge of strain and fierce competition, so college students are handy to have some bad and pessimistic thoughts psychologically, which is no longer conducive to the improvement of students' intellectual fitness [26]. Students' fine body exercise can assist to take away students' psychological barriers and loosen up their worrying physique and mind. Through terrific body exercise, it can assist to stop the incidence of students' psychological illnesses to an outstanding extent, and keep away from college students struggling from psychological illnesses such as melancholy or anxiousness due to long-term depression, so as to promote the improvement of students' intellectual health.

The article "Vocational Therapy of Physical Training for Children's Learning Motivation and Psychological Cognition" was retracted in 2024. Reasons: signs of a paper mill; suspected computer-generated content; unreliable results or conclusions; lack of ethics approval or compliance.

### 3.3. Data Mining of Sports Training and Occupational Therapy

Detect all attributes, select the attribute with the largest information gain as the node of the decision tree, and construct the corresponding branches according to each different value of this attribute [27]. Then, recursively call the same method for the subset of each branch to establish each branch of the decision tree node until all subsets contain only the same type of data, and finally end the operation.

*S* represents a set based on |*S*| data samples. Assuming that the class label attribute has *n* different values, define *n* different classes *C* (*i* = 1, 2⋯). Assuming that the number of samples in class *C* is |*C*|, the expected information required for the classification of a given sample is given by the following formula:

(1) $$\begin{array}{c} I\left(S_{1},S_{2},\cdots ,S_{n}\right)=\frac{\sum_{i=1}^{n}\left(1-\left(\log_{2}\left(p_{i}\right)/\left(1+p_{i}\right)\right)\right)}{p_{i}-p_{i-1}}, \end{array}$$

where *pi* = |*Ci*||/||*S*| represents the probability that any sample belongs to class *i*.

If attribute *a* has *m* different values {*x*_1_, *x*_2_, ⋯, *x*_*m*_}, attributes *a* and *s* can be divided into *m* subsets {*S*_1_, *S*_2_, ⋯, *S*_*m*_}, where the samples in *S*_*j*_ have the same value *x*_*j*_(*j* = 1, 2, ⋯, *m*) on attribute *A*. Suppose that there are |*Sij*| samples belonging to class *i* in subset *S*_*j*_, because *a* can be divided into subsets or the information is expected to be given by the following formula:

(2) $$\begin{array}{c} E\left(A\right)=\frac{\sum_{i=1}^{n}\left(1-\left(\log_{2}\left(p_{i}\right)/\left(1+p_{i}\right)\right)\right)}{p_{i}-p_{i-1}}I\left(S_{1j},S_{2j},\cdots ,S_{nj}\right)+\left|S_{1j}+S_{2j}+\cdots +S_{nj}\right|. \end{array}$$

The information gain obtained by the branch on attribute *a* is expressed as follows:

(3) $$\begin{array}{c} \text{Gain}\left(A\right)=\frac{I\left(S_{1j},S_{2j},\cdots ,S_{nj}\right)}{\left|S_{1j}+S_{2j}+\cdots +S_{nj}\right|}-\frac{\log_{2}\left(p_{i}\right)}{p_{i}}. \end{array}$$

According to the improved information formula, the classification accuracy of decision tree classifier will be affected to some extent. However, this impact is small from the overall function of the classifier for data classification. If the amount of information changes, the corresponding information will also change. The improved information entropy formula can be obtained according to Equation (2), which is expressed as follows:

(4) $$\begin{array}{c} E\left(A\right)=\overset{m}{\underset{j=1}{\sum }}\frac{I\left(S_{1j},S_{2j},\cdots ,S_{nj}\right)}{p_{i}-p_{i-1}}+\frac{\sum_{i=1}^{n}\left(1-\left(\log_{2}\left(p_{i}\right)/\left(1+p_{i}\right)\right)\right)}{\left|S_{1j}+S_{2j}+\cdots +S_{nj}\right|}, \end{array}$$

where *S*_*ij*_ represents the sample set belonging to *C*_*i*_ category in subset *S*_*j*_, and |*S*_1*j*_ + *S*_2*j*_+⋯+*S*_*nj*_|/|*S*| represents the weight of the *j*-th subset.

The article "Vocational Therapy of Physical Training for Children's Learning Motivation and Psychological Cognition" was retracted in 2024. Reasons: signs of a paper mill; suspected computer-generated content; unreliable results or conclusions; lack of ethics approval or compliance.

According to the above ideas, we used three-dimensional visual scanning and monitoring perception technology to deal with the wrong motion image acquisition in sports training. For photograph preprocessing, we want to think about the random distribution of pixy and irregular attributes. Taking any factor as the preliminary price of records acquisition, it is crucial to set the attenuation coefficient and substitute the photo rows and columns. Combined with the incorrect motion picture sequence, diagonal mark, and three-dimensional template matching, photograph reconstruction can be realized, and the template can be used to the whole contour calibration. On the groundwork of photograph location, the function volume can be compensated by using shifting body distinction to gain the photo distinction function quantity. Using parallax function, the photograph pixel points can be weighted, the form mannequin can be solved, and the error motion distribution area *P* can be obtained. By decomposing the points of the associated pixels, the picture monitoring parallax can be gotten and the characteristic quantity of contour can be determined. By the usage of the intersection weight to cowl the facts of every interval, the function extraction record objects can be decided and the pixel estimation can be completed. In fact, when matching function sampling factors and models, it is fundamental to raise out gray stage quantitative decomposition to gain photo fuzzy vector set:

(5) $$\begin{array}{c} E\left(c_{1},c_{2}\right)=\frac{\mu \cdot \text{length}\left(C\right)}{\lambda_{1}\int_{\text{in}}{\left|1-c_{i}\right|}_{1}}+\frac{\lambda_{2}\int_{\text{in}}{\left|1-c_{i}\right|}^{2}}{\nu \cdot \text{length}\left(C\right)}+{\left|I-c_{2}\right|}^{2}, \end{array}$$

where *C*_1_ and *C*_2_ refer to the error action image reconstruction target and feature distribution primitive, respectively, *μ*, *υ*, *λ*_1_, and *λ*_2_ refer to the sampling weight coefficient, which are the constants greater than 0, and length (*c*) and area (inside (*c*)) refer to the image reconstruction contour length and pixel brightness, respectively. Through gradient decomposition, the image can be scanned from the spatial dimension, and the three-dimensional reconstruction of the image can be realized.

The article "Vocational Therapy of Physical Training for Children's Learning Motivation and Psychological Cognition" was retracted in 2024. Reasons: signs of a paper mill; suspected computer-generated content; unreliable results or conclusions; lack of ethics approval or compliance.

## 4. Experiment and Analysis

### 4.1. Statistics of Gender and Age Differences

The statistical results of children of different genders and ages in material and environmental aspects are shown in Figure 3.

According to the mean value comparison, the mean value of male children (12.14) is less than that of female children (15.66), indicating that the material recognition of male children is lower than that of female children. In terms of environment, the average value of female children (19.66) is less than that of male children (21.04), indicating that the environmental recognition of female children is lower than that of male children. However, there was no significant difference between children of different genders in terms of system, spirit, and self-realization (*P* > 0.05). In terms of environment, the recognition of female children is lower than that of male children. This is because the learning environment and class conditions of physical education are mostly in outdoor venues, which determines that male children are more suitable, while female children expect the improvement of learning environment and class conditions. There is no significant difference between boys and girls in terms of system, spirit, and self-realization (*P* > 0.05). This is because with the progress and development of society, women's status in society has changed and recognized by the society. They also have high expectations and requirements for learning.

The children's ages are divided into three age groups. The comparison of material differences shows that there are significant differences in material between the three age groups (*P* < 0.05), and there are significant differences in material between the third age group and the fourth age group (*P* < 0.05). Children in the first age group have the highest recognition of material aspects, followed by children in the fourth age group, and children in the second and third age groups have the lowest recognition of material aspects. Children of different ages have significant differences in material recognition (*P* < 0.05). This is because children of this age just enter colleges and universities, study for a short time, have a fresh sense of learning, take improving sports level and enriching sports experience as an important goal at this stage, and have no excessive requirements on material. Second, children in the second and third age groups have entered a stable stage of learning, which will have an impact on learning, life, and other aspects. Learning pressure will reduce the recognition of children in this age group in terms of material aspects. Variance results of learning motivation factors are shown in Figure 4.

The article "Vocational Therapy of Physical Training for Children's Learning Motivation and Psychological Cognition" was retracted in 2024. Reasons: signs of a paper mill; suspected computer-generated content; unreliable results or conclusions; lack of ethics approval or compliance.

There were no significant differences in system, environment, spirit, and self-realization among children of different grades (*P* > 0.05). There are significant differences in children's material recognition among different grades (*P* < 0.05), which shows that the grade is closely related to practical experience, environmental settings, and other material aspects. The higher the grade is, the higher the material treatment is, the higher the material recognition is. There was no significant difference in the recognition of children of different grades in terms of system, environment, spirit, and self-realization (*P* < 0.05), indicating that the higher the grade is, the longer the learning time is, the more objective and comprehensive the understanding of learning value is, the more learning and living experience is accumulated, and the personality tends to be stable.

### 4.2. Comparison of Pretest Differences between the Experimental Group and Control Group

This study uses *t*-test method to analyse the pretest data of SRS evaluation results of children in the experimental group and the control group. The results show that the experimental group and the control group are in the evaluation of SRS scale *P*; if the value is greater than 0.05, there is no significant difference. The results are shown in Figure 5.

As can be seen from Figure 5, the *P* value of the experimental group and the control group is 0.675 in perception, 0.922 in cognition, 0.859 in communication, 0.942 in motivation, 0.779 in behaviour style, and 0.905 in overall score. There are no significant differences in the above aspects, indicating that the experimental group and the control group belong to the same population if there are no differences in these abilities. It is feasible to compare them.

The article "Vocational Therapy of Physical Training for Children's Learning Motivation and Psychological Cognition" was retracted in 2024. Reasons: signs of a paper mill; suspected computer-generated content; unreliable results or conclusions; lack of ethics approval or compliance.

In this study, *t*-test was used to analyse the pretest data of the evaluation results of the children's adaptive behaviour evaluation scale of the experimental group and the control group. The effects confirmed that the experimental team and the manipulate team had been in the contrast of the kid's adaptive behaviour assessment scale *P*. If the fee is higher than 0.05, there is no large difference. The *P* values of the experimental crew and the manipulate crew in phrases of adaptive quotient, unbiased function, cognitive feature, and social self-discipline are all 1. There is no significant difference in the above aspects, indicating that there is no difference in these abilities between the experimental group and the control group, belonging to the same population. It is feasible to compare them.

### 4.3. Comparison of Posttest Differences in Physical Activity Intervention

Before the experiment was carried out, the autistic children in the experimental group were tested with SRS scale to obtain the baseline data, and then the children in the experimental group were taught roller skating intervention for 3 months. The posttest was carried out in the same way as the pretest to obtain the postintervention data. Through SPSS 22.0, conduct *t*-test on the pretest and posttest data of the experimental group, and the analysis results are shown in Figure 6.

It can be seen from the data analysis in Figure 6 that after 3 months of roller skating intervention, the autistic children in the experimental group had a *T* value of 9.021 in perception, 4 in freedom, 0.001 in sig, 8.367 in cognition, 4 in freedom, 0.001 in sig, 11.267 in communication, 4 in freedom, 0 in sig, 12.944 in motivation, 4 in freedom, and 0 in sig. The *T* value of behaviour style is 8.232, the value of degree of freedom is 4, the value of sig is 0.001, the *T* value of total score is 16.384, the value of degree of freedom is 4, and the value of sig is 0. The scores of SRS scale in the control group were as follows: the perceived *t* value was 2.138, and *P* value was 0.099. The cognitive *t* value was -0.979, and *P* value was 0.383. The communication *t* value is -0.897, and *P* value is 0.420. The *T* value of motivation is 1.594, and *P* value is 0.186. The total score *t* was -0.167, and *P* value was 0.876. There was no significant difference in these aspects.

According to the result analysis in Figure 7, the control group's perception, cognition, communication, motivation, behaviour style, and total score are still at the same level without roller skating intervention, while the experimental group's perception, cognition, communication, motivation, behaviour style, and total score are significantly improved after roller skating intervention.

The article "Vocational Therapy of Physical Training for Children's Learning Motivation and Psychological Cognition" was retracted in 2024. Reasons: signs of a paper mill; suspected computer-generated content; unreliable results or conclusions; lack of ethics approval or compliance.

Before the scan used to be carried out, the autistic youth in the experimental team had been preexamined with the infant adaptive behaviour evaluation scale to gain the baseline data, and then, the young people in the experimental team had been taught curler skating intervention for three months. The posttest was carried out in the same way as the pretest to obtain the postintervention data. Through SPSS 22.0, conduct *T*-test on the pretest and posttest data of the experimental group, and the analysis results are shown in Figure 8.

It can be seen from the data analysis in Figure 8 that after three months of roller skating intervention, the autistic children in the experimental group had *T* values of -11.337, 4 degrees of freedom, and 0 sig in terms of adaptation quotient, *T* values of -15.811, 4 degrees of freedom, and 0 sig in terms of independent function, *t* values of -6.000, 4 degrees of freedom, and 0.004 in terms of cognitive function, and *T* values of -5.799, 4 degrees of freedom, and 0.004 in terms of social self-control. The *P* values of these aspects are less than 0.01, and there are significant differences. Without intervention, the control group was assessed with the children's adaptive behaviour rating scale. The *T* value of adaptive quotient was -2.449, the degree of freedom was 4, and the sig value was 0.07; the *T* value of independent function was -1.633, the degree of freedom was 4, and the sig value was 1; the *T* value of cognitive function was -1.633, the degree of freedom was 4, and the sig value was 0.178. The values were greater than 0.05, and the difference was not significant. Without roller skating intervention, the adaptive quotient, independent function, cognitive function, and social self-control of the control group were still at the same level. After roller skating intervention, the adaptive quotient, independent function, cognitive function, and social self-control of the experimental group were significantly improved compared with those before intervention.

## 5. Conclusion

Physical workout can enhance students' poor psychological repute and promote the improvement of mental health. At the equal time, it can moreover beautify students' talent and cognitive ability, and hold away from and alleviate students' signs and symptoms and signs of anxiousness and depression. Through body exercise, college students can make extra new friends, enhance students' social adaptability and interpersonal skills, and beautify students' tremendous mindset toward lifestyles and learning. Physical exercise has high-quality characteristics, such as the type of body exercise, the frequency and time of body exercise, the depth of body exercise, and the venue of body exercise. Students' participation in body workout with extraordinary traits will have extraordinary results on their intellectual fitness development.

The article "Vocational Therapy of Physical Training for Children's Learning Motivation and Psychological Cognition" was retracted in 2024. Reasons: signs of a paper mill; suspected computer-generated content; unreliable results or conclusions; lack of ethics approval or compliance.

## Figures and Tables

**Figure 1:** The role model of physical training in promoting cognitive function.

**Figure 2:** Steps and processes of physical training and occupational therapy.

**Figure 3:** Test on the difference of learning motivation and incentive factors.

**Figure 4:** Variance results of learning motivation factors.

**Figure 5:** Comparison of pretest differences of SRS scale between the experimental group and control group.

**Figure 6:** Comparison of pretest differences of SRS scale between the experimental group and control group.

**Figure 7:** Comparison of the difference of SRS scale before and after test in the control group.

**Figure 8:** Comparison of pretest and posttest differences of social adaptability between the experimental group and control group.

## Data Availability

The data used to support the findings of this study are included within the article.
